# An Unusual Presentation of Arteriovenous Malformation in a Pediatric Patient

**DOI:** 10.7759/cureus.4209

**Published:** 2019-03-09

**Authors:** Levonti Ohanisian, Angel Sidley, Joseph Wirth

**Affiliations:** 1 Internal Medicine, Florida Atlantic University Charles E. Schmidt College of Medicine, Boca Raton, USA; 2 Pediatrics, Florida Atlantic University Charles E. Schmidt College of Medicine, Boca Raton, USA; 3 Pediatrics, Nova Southeastern University School of Osteopathic Medicine, Plantation, USA

**Keywords:** arteriovenous malformations (avms), syncope, pediatrics

## Abstract

Arteriovenous malformations (AVMs) are defined as tortuous connections between arteries and veins that bypass the capillary system. Cerebral AVMs are rare with a general prevalence of 0.5%-1% with approximately one-fifth of these being diagnosed in infancy or childhood. Although most AVMs go undetected, the most common presenting symptom is hemorrhage. Despite a broad differential diagnosis for syncope described in the pediatric literature, there has been no report of AVM as the underlying etiology. We present a case of a seven-year-old female who presented with a single syncopal episode and was later found to have a large AVM involving mainly the thalamus on the right side and the basal ganglia with large intraventricular draining veins into the galenic venous system. To our knowledge, this is the only case reported of an AVM presenting as syncope in a pediatric patient.

## Introduction

Arteriovenous malformations (AVMs) are defined as tortuous connections between arteries and veins that bypass the capillary system resulting in hypertrophy of the arterial and venous components [1]. AVMs are considered to be of congenital origin [1] although cases of de novo AVM in pediatric patients have been described [2-3]. Cerebral AVMs are rare with a general prevalence of 0.5%-1% [4]. Of this, 18%-20% are diagnosed in infancy or childhood [4-5]. Although AVMs are most often undetected, hemorrhage is the most common clinical presentation of cerebral AVMs with recurrent seizure and headache being other presentations reported [1]. Despite the scarcity of AVMs in the pediatric population, the rate of hemorrhage observed is greater in this population as opposed to an adult population [4, 6] with a mean age of diagnosis at 31.2 years of age [7] and only 18%-20% of which are symptomatic under the age of 15 [4, 6]. Current treatment modalities include open vascular resection, radiosurgery, and endovascular embolization [1]. If left untreated, the overall risk of hemorrhage is between 2% and 4% in untreated cases [1].

Syncope in children has a reported incidence of 0.1%-0.5% [8-10]. The differential diagnosis for syncope includes vasovagal syncope (50%), orthostatic hypotension (20%), dehydration (15%), atypical seizure (7.5%), anemia (5%), migraine headache (5%), and minor head trauma (5%), as well as psychiatric causes and benign positional paroxysmal vertigo (BPPV) [8, 10]. Additionally, life-threatening causes such as long QT syndrome, hypertrophic cardiomyopathy, atrioventricular nodal reentry tachycardia, ventricular tachycardia, second-degree heart block that may result in sudden cardiac death and epilepsy may be underlying etiologies of syncope as a presenting symptom [10].

There have been cases described in the literature of adult patients with AVM who have presented with syncope [11-12]. To our knowledge, there has been no case in the literature that describes syncope as the presenting symptom of AVM in a pediatric patient. We present the case of a seven-year-old female who presented with syncope secondary to AVM. This highlights the importance of including AVM in the differential diagnosis of syncope in the pediatric population.

## Case presentation

A seven-year-old female with no significant past medical history initially presented with a syncopal episode while at a birthday party, with loss of consciousness for 2-3 seconds and mild upper body stiffness without a postictal state. The patient reportedly was on the swing at a local park when she experienced her syncopal episode. As per her mother, who watched the entire episode, she did not fall off the swing and immediately returned to normal activity. The patient had no prior history of syncope, headaches, seizures, vomiting, diplopia, or blurry vision, and no family history of seizure disorder, cardiac abnormality, CNS disorder, or AVM. Upon follow up with her pediatrician the next day, the patient was alert, happy, and in no apparent distress. A comprehensive physical exam performed including extensive neurological examination was unremarkable.

Despite this, the pediatrician chose to order a head CT to rule out intracranial pathology, as well as a CBC with differential, CMP, thyroid profile, 2D echo with doppler of the heart, and 12-lead electrocardiogram. All her laboratory results were within normal limits. Head CT revealed marked abnormality to the thalamus, lateral ventricle, and the periventricular area on the right side extending into the foramen of Monroe and causing hydrocephalus. Based upon this, a differential diagnosis including brain tumor, AVM, and neurofibromatosis was developed.

At this point, the pediatrician ordered an MRA that showed an AVM. The patient was subsequently sent for an MRI of the brain with gadolinium which revealed hydrocephalus and a large AVM involving mainly the thalamus on the right side and the basal ganglia with large intraventricular draining veins into the galenic venous system (Figure 1). The size of the malformation was noted to be 5 cm x 4 cm x 3 cm. There were no signs of intracranial hemorrhage. Cerebral angiogram confirmed these findings (Figure 2).

**Figure 1:** MRI with gadolinium. MRI with gadolinium demonstrating a 5 cm x 4 cm x 3 cm arteriovenous malformation involving mainly the thalamus on the right side and the basal ganglia with large intraventricular draining veins into the galenic venous system.

**Figure 2:** Cerebral angiogram. Cerebral angiogram showing a large right basal ganglia and thalamic arteriovenous malformation with mild involvement of the left basal ganglia.

Three subsequent neurosurgical evaluations demonstrated an unremarkable neurological examination with no asymmetries on cranial nerve examination, strength, muscle tone, or reflexes. Her sensory and cerebellar examinations were within normal limits as well, and the neurologist concluded that the AVM was not associated with any neurological deficits and no symptoms referable to the ventricular obstruction. An EEG obtained showed no abnormalities. An ophthalmology consult demonstrated a normal ophthalmological examination with no evidence of AVM in the retina. Due to the AVM size and structural involvement, surgery was ruled out as a possible course of treatment. All neurosurgical consults concluded that the patient should receive routine imaging every six months to ensure no change in size and bleeding status. A repeat MR angiogram (Figure 3) and MRI eight months after the original confirmed no increase in overall size of the vascular malformation. The patient was routinely monitored with follow up CT and MRI scans every six months for the next six years, which demonstrated no change in size of her AVM and no evidence of bleeding. The patient also exhibited no signs of neurological deficit, and never experienced a repeat syncopal episode during this time. She was then lost to follow up and passed away as a result of AVM rupture 12 years after presentation.

**Figure 3:** MR angiogram. MR angiogram corroborating findings of cerebral angiography.

## Discussion

Arteriovenous malformations are considered embryological in origin and as the result of arteriovenous shunting due to a tortuous direct connection between arteries and veins that results in hypertrophy of the arterial and venous components of the AVM [1]. Although the exact pathophysiological mechanism has not been elucidated, it is postulated that the abnormality occurs during the third week of embryogenesis [1]. Cerebral AVMs are rare in children with a prevalence of 0.5%-1% [5] with hemorrhage being the most common clinical manifestation of cerebral AVM [4]. Other presentations include recurrent seizures and headache [1]. A multicenter prospective study aimed at describing characteristics of AVMs involved 1289 consecutive patients and concluded that the mean age of diagnosis is 31.2 years of age with AVM diameter being under 3 cm in 38% of cases [7].

Syncope is defined as a transient loss of consciousness and postural tone due to cerebral hypoperfusion [10]. The incidence of syncope in children is postulated to be between 0.1% and 0.5% [10]. The differential diagnosis of syncope in children and adolescents as discussed in a retrospective review of 77 patients includes vasovagal syncope (50%), orthostatic hypotension (20%), dehydration (15%), atypical seizure (7.5%), anemia (5%), migraine headache (5%), and minor head trauma (5%) [8]. The authors concluded a limited routine evaluation is sufficient for children presenting with syncope as most are caused secondary to vasovagal syncope, however, acknowledged that life-threatening causes exist and further outcome-based studies are needed to validate this recommendation [8]. Investigations since have replicated similar study designs and elaborated on underlying life-threatening complications that manifest as syncope. One such study involving 268 pediatric patients with a mean age of 12 concluded that careful medical evaluation including hospital admission is necessary for patients presenting with syncope as it may be the first finding of underlying cardiac or neurological disease such as long QT syndrome, hypertrophic cardiomyopathy, atrioventricular nodal reentry tachycardia, ventricular tachycardia, second-degree heart block that may result in sudden cardiac death and epilepsy [10]. Interestingly, 82.1% of patients experienced recurrent syncope and in addition to known causes, the authors mentioned psychiatric causes and BPPV as rare but additional etiologies [10].

There have been reports of adults with AVMs presenting with recurrent syncopal episodes. De Biase et al. reported a case of recurrent episodes of syncope in a 66-year-old patient with cerebral AVM suggestive of an epileptogenic mechanism [11]. Carboni and Quattrocchi describe another case of long-term syncope in a 73-year-old male with AVM found on brain MRI [12]. To our knowledge, there has been no report of syncope as the initial presentation of AVM in the pediatric population. We present a pediatric case of syncope caused by AVM possibly secondary to an epileptogenic mechanism. Our case illustrates the importance of including AVM as a life-threatening cause of syncope in the pediatric population.

## Conclusions

This case illustrates that abnormal physical examination and laboratory findings should not be required to justify imaging studies to exclude intracranial pathology, particularly when there is no identifiable etiology of syncope. Additionally, our case suggests that AVM should be included in the differential diagnosis of syncope in a pediatric patient.
